# A New ELECTRE Method Based on Left and Right Score for Multicriteria Decision-Making

**DOI:** 10.1155/2023/6414686

**Published:** 2023-11-10

**Authors:** Faeze Jokar, M. Jalali Varnamkhasti, A. Hadi-Vencheh

**Affiliations:** Department of Mathematics, Isfahan (Khorasgan) Branch, Islamic Azad University, Isfahan, Iran

## Abstract

The procedure for ranking the performance of systems using the method Elimination and Choice Translating Reality (ELECTRE) is one of the most important and practical methods in multicriteria decision-making (MCDM). The classical ELECTRE technique uses the concept of dominance implicitly. In this method, all options are evaluated using a comparison of unexpected rankings, thus eliminating ineffective options. All stages of the electrification technique are based on a coordinated set and an uncoordinated set, which is why it is known as “coordination analysis.” The ELECTRE method has two important weaknesses, first, the use of thresholds, which are used to calculate the coordination and noncoordination matrix, and second, this method does not give us a complete and final ranking and is limited to the top options. In order to reduce these weaknesses in this research, interval fuzzy numbers have been used. In the proposed process, the numbers to the left and right of the intervals are considered, and a better method is presented with fuzzy techniques based on the ELECTRE technique. In the research results, using the examples taken from previous researches, the ability of the proposed method is shown.

## 1. Introduction

Choosing the best project is a multicriteria decision-making (MCDM) issue that includes both quantitative and qualitative criteria. In many cases, finding the exact value for a project such as the best performance, best structure may be very difficult or impossible in practice [1]. In these problems, in most cases, the value of the choices is proportional to the criteria, and the weight of the criteria is fuzzy numerical, so numerical contracts to solve the problems of choice and MCDM problems in general have a vague and linguistic personality. In this case, fuzzy MCDM methods are used to solve these problems [2, 3].

Today, there is extensive competition for economic problems and relations that are effective on them including production or constant services on the markets. Under the circumstances and in order to save the companies and keeping them competitive, companies have to pay attention to methods that gain maximum results and increase production and services and have real function. Multicriteria decision-making is being used for risk assessment and choosing replacements that compete with more than one criterion. One of the most significant and useful processes in multicriteria decision-making is the strategy known as “elimination by choice” (translating reality) for ranking the performance of systems. The traditional elimination by choice: translating reality method implicitly makes use of dominance. This approach compares unexpected ranks to evaluate each choice, weeding out the inefficient ones. The electrification technique is known as “coordination analysis” since it is based on a coordinated set and an uncoordinated set at each stage. There are two significant flaws in the elimination by choice: translating reality approach. First, the coordination and noncoordination matrix is calculated using thresholds. Second, this approach just considers the top choices and does not provide a comprehensive or final rating [4]. On the other hand, one of the multicriteria decision-making methods that were used in different fields is the ELECTRE method. In this method, alternative choices are analyzed by interval comparisons; therefore, ineffective choices will be eliminated. All steps of the ELECTRE method are based on harmonic and inharmonic sets and thus are called harmonic analysis. In other words, the concept of dominance is being used implicitly. Herein, choices will be compared dually, and then, weak choices will be eliminated. After the ELECTRE I procedure, other versions of this technique (ELECTRE II-V, A) were introduced and used. The ELECTRE process was first proposed by Roy in 1968 [5] for solving MCDM problems. Main ideas of the ELECTRE method first published as a research report in 1966. ELECTRE method II Roy [6] is the closest method to ELECTRE I in the family, and their difference is in the definition of two prioritizing relations instead of one in ELECTRE I. In ELECTRE II, there could be strict or weak preferences for a choice. Therefore, the intensity of preference is clearly explained in the ELECTRE II method. However, in the ELECTRE 1 method, indifference or strict preference of a choice over the other one is being discussed, and the intensity of preference is not explained. Due to the high sensitivity of the preference threshold and considering the different relationships between the choices in the ELECTRE II method, favorable results were not obtained in solving the problems, therefore, to solve these problems, the methodELECTRE III were replaced.. In other words, ELECTRE III is similar to ELECTRE II and also adds examined extraversion relations and uses pseudocriteria, and these are features that use priority and indifference thresholds [6]. The important point about the ELECTRE IV method is that there is no need for weights for determining criteria which is a step against mentality. Interpreting this lack of weight is similar to the ELECTRE I method “all criteria are not equally important, but none of them have low values in their relations with others.” [7]

The ELECTRE-TRI model is a member of the ELECTRE multicriteria methods family for ranking which has been proposed by Yu [8] for the first time and then developed in later years. This method is for multicriteria decision-making that choices are classified based on predetermined intervals. This classification is the result of the compassion of choices with profiles that represent the boundary of beds. In cases that data are incomplete, another method will be which is called ELECTRE-IS. One of the important ELECTRE method defects is measuring performance and weight criteria. In reality, it is not always possible to present an explicit value for the choices and the criteria [9]. The fuzzy sets theory is an ideal and appropriate method for solving these problems. Fuzzy logic is being used for explaining linguistic and vague variables [10]. Therefore, ELECTRO FUZZY method was made by using fuzzy techniques in the ELECTRE method. ELECTRO FUZZY is used for solving many problems in real life along with MCDM methods [11]. By comparing these methods, it is observed that ELECTRO FUZZY methods had a better performance in solving real-life problems and real events where events are often presented in qualitative and linguistic terms. In this method, few input data are needed for a lot of choices and criteria, and their performance can be analyzed easily, and there is no obligation to binary comparisons [12].

Over the years, extensive research on ELECTRE family methods has emerged, and this method has shown different applications. Also, by using hybrid methods such as fuzzy sets, interval fuzzy, gray numbers, and the like with the ELECTRE method, the popularity of this method in MCDN problems increased [13, 14]. Kumar et al. [15] were trying to create a framework for analyzing the operational performance of cellular mobile telephone service providers (CMTSP) in Delhi, India. The studies are done by using a fuzzy ELECTRE method for comparing the performance of cellular mobile telephone service providers. Data analyzation is done by the Telecom Regulatory Authority of India (TRAI). Adeel et al. [16] in their research introduced a multipolar fuzzy method with a new suffix of ELECTRE-1 for solving multicriteria decision-making based on multipolar fuzzy sets and claimed that it is a strong tool for indicating inaccuracy and unreliability in multipolar data. The proposed technique is more flexible and practical in the real world, especially when the data are the result of multipolar information. In the proposed method, alternative ranking is being evaluated by mental criteria, and its normal weights are assessed by the decision-maker. Then, numerical examples are presented to prove the feasibility, validity, and effectiveness of the proposed method. Singh & Kaushik [17] studied intrusion detection system (IDS) and automated intrusion response system (AIRS). Since intrusion detection system detects attacks and generates alerts while an automated intrusion response system (AIRS) chooses the appropriate response from response sets based on some response choice criteria and helps reducing infiltration without delay, therefore, the main challenges for designing AIRS are the accurate measuring of the weight, importance of each response choice criterion, and prioritizing a set of intrusion response. These researchers used fuzzy ELECTRE method in their study. In conclusion, by using this technique, they showed prioritization of a prioritized response set can be used more by each AIRS model for automatic selection of an appropriate response to counter attacks based on given criteria. Kumar [18] studied recruiting competition. This research addresses the issue of recruiting personnel for international safe company sales engineer. The recruiting criteria were obtained through analysis conducted by human resource company and study specific literature, and best candidate is chosen by evaluating five criteria by three decision-makers and by using fuzzy ELECTRE method.

Qu et al. [19] presented a three-step MCDM method considering the best-worst method based on time interval. In the three-step method, the weight of experts, the weight of criteria, and the weighted sum process in social networks were considered. The proposed MCDM model is innovative in a situation where both the weight of the experts and the criteria are unknown and provides mathematical models to solve them, respectively. Finally, a case is used to prove the usefulness and availability of the new MCDM method. The results show that the new MCDM approach can not only reduce decision-making mentality but can also effectively solve MCDM problems. Suo et al. [20] in their research, in order to reduce the computational complexity on fuzzy sets with open value, they proposed the concept of fuzzy set with value of polygonal intervals. In this research, it has been shown that fuzzy numbers with a value of polygon interval *n* can approximate fuzzy numbers of general value with any accuracy. The results also show that the arithmetic operations introduced here are continuous on *n* fuzzy numbers with polygon interval values. Rodrigues et al. [21] in their research presented an algorithm that could provide a combination of parameters for ELECTRE II, III, or IV methods. In their work process for selecting the parameters, they used the technique of the machine learning set, random forest, and called it the ranking tree algorithm. Mohammadghasemi et al. [22] considered the choice of material handling equipment as a multicriteria set and then a version of type-2 fuzzy sets called Gaussian-type fuzzy sets as an alternative to traditional triangular membership functions for weights and sizes in Commented. In order to show the proper performance of this method, in a real case study and an illustrative example, the method was implemented. Then, the ranking results were compared with other results in the literature, and finally, the sensitivity analysis to show the strength and stability of the results showed the very good performance of the proposed method.

According to the study of Türk et al. [23], a multicriteria decision method based on interval fuzzy set is selected to select the best location for electric charging stations. In this method, it is improved by simulated annealing, which achieves the best configuration of the parameters of interval membership functions with two different aggregation operators. The results show that this approach actually improves the model, better showing the related uncertainties embedded in the membership functions of the interval, which leads to a more efficient fuzzy system. Jeevaraj [24] first introduced fuzzy sets of spaced formats and performs some mathematical operations on the IVFFS class. In the second step, he introduced the different scoring functions in the IVFFS class and examines their properties. Third, he compared different ranking methods with the proposed score functions to show the performance of the proposed score functions. Mokhtarian and Hadi Vancheh [25] in their research addressed the issue of selecting the location of facilities from among alternative locations and proposed a new method of fuzzy TOPSIS from fuzzy methods according to the left and right scores.

In this study, the left and right intervals are used for the ELECTRE technique. In fuzzy MCDM problems (normal fuzzy numbers), ranking choices are done in terms of criteria which in most of problems, ranking of criteria is numbers between [0, 1] that is a difficult task to do. Under the circumstance, choices ranking is in terms of criteria (weight of criteria), and interval–amount numbers will be used. Amount of best choice is necessarily the farthest distance to the worst option and the closest distance to the best option. On the other hand, the interval method has some problems such as being single abelian and having an interval dependence. So, we try to improve the rankings by using the ELECTRE method. In the ELECTRE method, we compare options to criteria. All previous methods have been one dimensional; however, ELECTRE is a method that we compare each of options to each criterion. On the other hand, interval method is a dependent method; therefore, ELECTRE method obviates this dependency and makes interval method more practical. Fuzzy method introduces the concept of maximizing the set and minimizing the set for determining sorting value of each fuzzy number based on left and right numbers and uses these values to determine the fuzzy numbers. In this method, options are compared dually, and the dominant and weak options are identified, and then, the weak options are removed. In this paper, we proposed a method for solving interval-fuzzy MCDM problems to solve this problem as much as possible and rank the options using this method. Here, we are trying to extend the method of ELECTRE by using terms of compatibility and mismatch and apply a new idea to solve such problems. So, we are trying to express the idea of resolving compatibility and incompatibility problems.

In short, it can say ELECTRE is one of the decision-making methods that compared with several multicriteria decision-making techniques. Furthermore, it requires significant amount of primary data. ELECTRE method has a difficulty that it needs precise measurements of performance ratings and criteria weights. Scoring or assigning a number to an action is very weak, so it may confuse to get the real result. In this point of view, it is needed to eliminate also two basic disadvantages: first, the use of thresholds, which are used to calculate the coordination and noncoordination matrix; second, this method does not give us a complete and final ranking and is limited to the top options. In order to reduce these weaknesses in this research, the idea of using interval fuzzy numbers is presented.

In the continuation of this article, the definitions and relations of fuzzy logic will be discussed first. Then, the ELECTRE method and fuzzy ELECTRE with new technique will be presented. At the end, the new model is checked with some numerical examples, and the obtained results are analyzed.

## 2. Theory of Fuzzy Sets

Fuzzy sets are a more general case of ordinary sets and were introduced for the first time by Zadeh [26] and are a solution for showing the inaccuracy and ambiguity in real world. A fuzzy set is a set of objects in a reference set of information where the boundary is a vague reference set (its boundary is not clear). Each fuzzy set is determined by a membership function and assigned each member of the reference set a number in the interval (0, 1). The assigned value is the membership rate which show to what extent the relevant member belongs to the set (the larger the number, the larger the set it belongs to). If the assigned value is zero, the member does not belong to the set. But if the assigned value is one, the member is wholly owned by the set, and if the assigned value is a number in the open interval (0, 1), to some extent that member belongs to the set. Therefore, each fuzzy set is completely specified by its membership function. Suppose *X* is a reference set.

An A˜ fuzzy set from A fuzzy set is called convex only if we have this condition for *X*1 & *X*2 of *X*:

(1) $$\begin{array}{c} \mu \tilde{A}\left(\lambda X1+\left(1-\lambda \right)X2\right.\geq \min\left(\mu \tilde{A}\left(X1\right),\mu \tilde{A}\left(X2\right)\right.\text{.} \end{array}$$

We call a fuzzy set normal if there is a *X* that its membership degree is one. Fuzzy numbers are a special case of fuzzy sets which are both normal and convex that are given by an interval of real numbers that each of them are shown with a membership degree between (1, 0). Most common fuzzy numbers are triangular and trapezoidal fuzzy numbers that their membership function is defined as follows:

(2) $$\begin{array}{c} \mu_{\tilde{A}}\left(X\right)=\left\{\begin{array}{c} \begin{array}{cc} \frac{\left(x-a\right)}{\left(b-a\right)}, & a\leq x\leq b, \end{array}\\ \begin{array}{cc} \frac{\left(d-x\right)}{\left(d-b\right)}, & b\leq x\leq d, \end{array}\\ \begin{array}{cc} 0, & otherwise, \end{array} \end{array}\right.\\ \mu_{\tilde{A}}\left(X\right)=\left\{\begin{array}{c} \begin{array}{cc} \frac{\left(x-a\right)}{\left(b-a\right)}, & a\leq x\leq b, \end{array}\\ \begin{array}{cc} 1, & b\leq x\leq c \end{array}\text{,}\\ \begin{array}{c} \begin{array}{cc} \frac{\left(d-x\right)}{\left(d-c\right)}, & c\leq x\leq d, \end{array}\\ \begin{array}{cc} 0, & otherwise. \end{array} \end{array} \end{array}\right. \end{array}$$

For simplicity, triangular and rectangular numbers are shown with (*a*, *b*, *c*) & (*a*, *b*, *c*, *d*) where *b*=*c*, suppose *A˜* = (*a*_1_, *a*_2_, *a*_3_) & $\tilde{B}=\left(b^{1},b^{2},b^{3}\right)$ are two triangular fuzzy numbers; then,

(3) $$\begin{array}{c} \tilde{A}+\tilde{B}=\left(a_{1}+b_{1},a_{2}+b_{2},a_{3}+b_{3}\right)\text{,}\\ \tilde{A}-\tilde{B}=\left(a_{1}-b_{3},a_{2}-b_{2},a_{3}-b_{1}\right)\text{,}\\ \tilde{A}\times \tilde{B}=\left(a_{1}.b_{1},a_{2}.b_{2},a_{3}.b_{3}\right)\text{,}\\ \tilde{A}÷\tilde{B}=\left(\frac{a_{1}}{b_{3}}.\;\frac{a_{2}}{b_{2}}.\frac{a_{3}}{b_{1}}\right)\text{.} \end{array}$$

Concerning the normalization process, triangular numbers are suggested as follows:

(4) $$\begin{array}{c} \left({\left(a_{ij}\right)}_{N},{\left(b_{ij}\right)}_{N},{\left(c_{ij}\right)}_{N}\right)=\left(\frac{a_{ij}-a_{j}^{\min}}{{∆}_{\min}^{\max}},\frac{b_{ij}-a_{j}^{\min}}{{∆}_{\min}^{\max}},\frac{c_{ij}-a_{j}^{\min}}{{∆}_{\min}^{\max}}\right),i=1,\ldots ,n\text{.} \end{array}$$

If the criteria are the profit criteria (positive criteria), we will do as follows:

(5) $$\begin{array}{c} \left({\left(a_{ij}\right)}_{N},{\left(b_{ij}\right)}_{N},{\left(c_{ij}\right)}_{N}\right)=\left(\frac{a_{ij}-a_{j}^{\min}}{{∆}_{\min}^{\max}},\frac{b_{ij}-a_{j}^{\min}}{{∆}_{\min}^{\max}},\frac{c_{ij}-a_{j}^{\min}}{{∆}_{\min}^{\max}}\right),i=1,\ldots ,n\text{.} \end{array}$$

If the criteria are expenditure (negative criteria), we will do as follows:

(6) $$\begin{array}{c} C_{j}^{\max}=\max C_{ij},where\;i=1,\ldots ,n\text{.} \end{array}$$

This is the case for a triangle number, if the number is trapezoidal to normalize it: (profit criteria)

(7) $$\begin{array}{c} {\left({\tilde{y}}_{ij}\right)}_{N}=\left({\left(a_{ij}\right)}_{N},{\left(b_{ij}\right)}_{N},{\left(c_{ij}\right)}_{N},{\left(d_{ij}\right)}_{N}\right)=\left(\frac{a_{ij}-a_{j}^{\min}}{{∆}_{\min}^{\max}},\frac{b_{ij}-a_{j}^{\min}}{{∆}_{\min}^{\max}},\frac{c_{ij}-a_{j}^{\min}}{{∆}_{\min}^{\max}},\frac{d_{ij}-a_{j}^{\min}}{{∆}_{\min}^{\max}}\right)\text{.} \end{array}$$

Expenditure criteria are as follows:

(8) $$\begin{array}{c} \left({\left(a_{ij}\right)}_{N},{\left(b_{ij}\right)}_{N},{\left(c_{ij}\right)}_{N},{\left(d_{ij}\right)}_{N}\right)=\left(\frac{d_{ij}-d_{j}^{\max}}{{∆}_{\max}^{\min}},\frac{b_{ij}-a_{j}^{\min}}{{∆}_{\max}^{\min}},\frac{c_{ij}-a_{j}^{\min}}{{∆}_{\max}^{\min}},\frac{d_{ij}-a_{j}^{\min}}{{∆}_{\max}^{\min}}\right)\text{,} \end{array}$$

where

(9) $$\begin{array}{c} d_{j}^{\max}=\max d_{ij}\text{,}\\ a_{j}^{\min}=\min a_{ij}\text{,}\\ \Delta_{\min}^{\max}=d_{j}^{\max}-a_{j}^{\min}\text{,}\\ \Delta_{\max}^{\min}=a_{j}^{\min}-d_{j}^{\max}\text{.} \end{array}$$

Since the proposed method is based on the left and right fuzzy numbers, in the following section, the concept of left and right fuzzy numbers will be explained. Left and right numbers are first introduced by Chen [27]. Suppose k˜ is the fuzzy number, its left and right numbers are defined as follows [27]:

(10) $$\begin{array}{c} {\left(l_{s}\right)}_{\tilde{k}}={sup}_{x}\;\left[\mu_{\tilde{k}}\left(x\right)\wedge \mu_{\min}\left(x\right)\right]{\left(R_{s}\right)}_{\tilde{k}}={sup}_{x}\;\left[\mu_{\tilde{k}}\left(x\right)\wedge \mu_{\max}\left(x\right)\right]\text{.} \end{array}$$

And the membership function for the minimum set and the maximum set for each fuzzy number is as follows:

(11) $$\begin{array}{c} \mu_{\max}\left(x\right)=\left\{\begin{array}{cc} x\text{,} & \;0\leq x\leq 1\text{,}\\ 0\text{,} & otherwise\text{,} \end{array}\right.\\ \mu_{\min}\left(x\right)=\left\{\begin{array}{cc} 1-x\text{,} & 0\leq x\leq 1\text{,}\\ 0\text{,} & otherwise\text{.} \end{array}\right. \end{array}$$

To put it simply and for determining normalized left and right numbers of fuzzy numbers, we define equations ${\tilde{y}}_{ij}$ as follows:

(12) $$\begin{array}{c} {\left(l_{s}\right)}_{ij}=\frac{{\left(b_{ij}\right)}_{N}}{1+{\left(b_{ij}\right)}_{N}-{\left(a_{ij}\right)}_{N}}\text{,}\\ {\left(R_{s}\right)}_{ij}=\frac{{\left(c_{ij}\right)}_{N}}{1+{\left(c_{ij}\right)}_{N}-{\left(b_{ij}\right)}_{N}}\text{.} \end{array}$$

For trapezoidal,

(13) $$\begin{array}{c} {\left(l_{s}\right)}_{ij}=\frac{{\left(b_{ij}\right)}_{N}}{1+{\left(b_{ij}\right)}_{N}-{\left(a_{ij}\right)}_{N}}\text{,}\\ {\left(R_{s}\right)}_{ij}=\frac{{\left(d_{ij}\right)}_{N}}{1+{\left(d_{ij}\right)}_{N}-{\left(c_{ij}\right)}_{N}}\text{.} \end{array}$$

### 2.1. ELECTRE Technique

ELECTRE method (ELimination and Choice Expressing REality method) is one of most famous ranking methods. In this method, options are compared dually, and the dominant and weak options are identified, and then, the weak options are removed. In a multicriteria decision-making problem, *n* is the criterion, and *m* is the option, to choose the best option by ELECTRE method, and the following steps should be taken [1, 2]:

Step 1: creating a decision matrix
Based on the number of criteria, the number of options, and the evaluated values of the options, the following decision matrix is created for different criteria:
  (14) $$\begin{array}{c} X=\left[\begin{array}{ccc} x_{11} & \cdots & x_{1n}\\ \vdots & \ddots & \vdots \\ x_{m1} & \cdots & x_{mn} \end{array}\right]\text{,} \end{array}$$
where *x*_*ij*_ is the function of option *i*(*i* = 1,…, *m*) in relation with criterion *j*(*j* = 1,…, *n*).
Step 2: descaling decision matrix:
At this stage, dimensions with different dimensions are transformed into dimensionless criteria, and matrix *R* is defined as follows:
  (15) $$\begin{array}{c} R=\left[\begin{array}{ccc} r_{11} & \cdots & r_{1n}\\ \vdots & \ddots & \vdots \\ r_{m1} & \cdots & r_{mn} \end{array}\right]\text{.} \end{array}$$
There are different methods for descaling, but in ELECTRE method, the following equation is used:
  (16) $$\begin{array}{c} r_{ij}=\frac{x_{ij}}{\sqrt{x_{ij}^{2}}}\text{.} \end{array}$$
Step 3: determining weight of criteria
At this stage, considering the significance coefficients of different criteria in decision-making, the significance coefficient of criteria is defined as follows:
  (17) $$\begin{array}{c} W=\left[W_{1}W_{2}\ldots W_{n}\right]. \end{array}$$
Elements of vector “*W*” are significance coefficients of the criteria
Step 4: determining weighted normalized matrix
The weighted decision matrix is obtained by multiplying the descaled decision matrix in the criteria weighting vector
  (18) $$\begin{array}{c} v_{ij}=w_{j}r_{ij},i=1,\ldots ,m\;and\;j=1,\ldots ,n\text{.} \end{array}$$
Step 5: forming a set of concordance and discordance criteria
For each pair of options *k*, *e*, (*k*, *e* = 1,2,…, *m*, *j* = 1,…, *n*) are divided into *Pro* and
*Cons* subsets. *Pro* criteria set is defined as follows for positive and negative criteria:
  (19) $$\begin{array}{c} S_{ke}=\left\{j|v_{kj}\geq v_{ej}\right\}\text{,}\\ S_{ke}=\left\{j|vkj\leq v_{ej}\right\}\text{.} \end{array}$$
*Cons* criteria set is defined as follows for positive and negative criteria:
  (20) $$\begin{array}{c} I_{ke}=\left\{j|v_{kj}\;<\;v_{ej}\right\}\text{,}\\ I_{ke}=\left\{j|v_{kj}\;<\;v_{ej}\right\}\text{.} \end{array}$$
Step 6: creating concordance matrix
The concordance matrix is a square matrix which its dimension is the number of options. Each of the elements of this matrix is called the index of concordance between two options. In other words, to calculate the index of concordance of *k*, *e* options should be compared, and its value is the sum of the weightings of the criteria that option *k* has in proportion to option *e*. In mathematical terms, the index of concordance is calculated from the following equation:
  (21) $$\begin{array}{c} C_{ke}=\frac{\sum_{j\epsilon s_{ke}}w_{j}}{\sum_{j=1}w_{j}}\text{.} \end{array}$$
The index of concordance indicates the degree of superiority that option *k* has over option *e*, and the value varies from zero to one. By calculating the index of concordance for all the pairs of options, one can define the concordance matrix as follows, and in general, this matrix is not symmetrical.
  (22) $$\begin{array}{c} C_{ke}=\underset{j\epsilon s_{ke}}{\sum }w_{j}\text{.} \end{array}$$
Step 7: determining discordance matrix
Discordance matrixis a square matrix which its dimension is the number of options. Each of the elements of this matrix is called the index of disagreement of these two options. The value of this index is calculated as follows [23]:
  (23) $$\begin{array}{c} d_{ke}=\frac{\max_{j\epsilon I_{ke}}\left|v_{kj}-v_{ej}\right|}{\max_{j\epsilon J}\left|v_{kj}-v_{ej}\right|}\text{.} \end{array}$$
The value of disagreement index varies from zero to one. By calculating the index of disagreement for all pair of options, the discordance matrix can be defined as follows. In general, this matrix is not symmetrical.
  (24) $$\begin{array}{c} D=\left[\begin{array}{ccc} - & d_{12}\cdots & d_{1m}\\ d_{21} & - & d_{2m}\\ d_{m1} & d_{m\left(m-1\right)}\cdots & - \end{array}\right]\text{.} \end{array}$$
The information in concordance matrix has major differences from the information in the discordance matrix, and in fact, this information is complimentary. Differences between weights are obtained by the concordance matrix, whereas the difference between specified values is obtained by the discordance matrix.
Step 8: creating concordance dominance matrix
In step 6, it was expressed how to calculate concordance. At this point, a certain value is specified by the index of concordance, which is called the threshold of concordance and is denoted by $\bar{C}$. The concordance threshold is obtained by averaging the agreement indices (the matrix elements of the agreement). In mathematical terms, the amount of concordance threshold is calculated from the following equation:
  (25) $$\begin{array}{c} \bar{C}\overset{m}{\underset{k=1}{\sum }}\overset{m}{\underset{e=1}{\sum }}\frac{C_{ke}}{m\left(m-1\right)}\text{.} \end{array}$$
Concordance dominance matrix (*f*) is created based on the amount of concordance threshold. If it is greater than $\bar{C}$ option *k* superiority over option, *e* is acceptable; otherwise, option *k* has no advantage over option *e*. Thus, the elements of the concordance dominance matrix are calculated by the following equation:
  (26) $$\begin{array}{c} f_{ke}=\left\{\begin{array}{cc} 1\text{,} & C_{ke}\geq \bar{C}\text{,}\\ 0\text{,} & C_{ke}<\bar{C}\text{.} \end{array}\right. \end{array}$$
Step 9: creating discordance dominance matrix
The discordance dominance matrix (*G*) is formed as the concordance dominance matrix. For this purpose, the discordance threshold $\bar{d}$ is calculated from the averaging of the discordance indices (discordance matrix elements).
  (27) $$\begin{array}{c} \bar{d}=\overset{m}{\underset{k=1}{\sum }}\overset{m}{\underset{e=1}{\sum }}\frac{d_{ke}}{m\left(m-1\right)}\text{.} \end{array}$$
As stated in step 7, the lower the value of the opposition index, the better it is. Because it shows the superiority of option *k* over *e*. Therefore, the elements of the discordance dominance matrix *G* are calculated as follows:
  (28) $$\begin{array}{c} g_{ke}=\left\{\begin{array}{cc} 1\text{,} & d_{ke}\leq \bar{d,}\\ 0\text{,} & d_{ke}>\bar{d.} \end{array}\right. \end{array}$$
Step 10: creating final dominance matrix
The final dominance matrix *H* is obtained by multiplying each of the dominance matrix elements of *F* by its corresponding elements in the discordance dominance matrix *G*.
  (29) $$\begin{array}{c} h_{ke}=f_{ke}g_{ke}. \end{array}$$
Step 11: choosing the best option

The final dominance matrix *H* gives a detailed description of options. For example, if the value of ℎ is equal to one, it means that the superiority of the option *k* over *e* is acceptable in both concordance and discordance cases (i.e., its advantage is greater than the threshold of concordance, and its disagreement or its weakness is lower than the threshold of discordance). However, the option *k* still has the chance to be dominated by other options. An option should be chosen that is more dominant than being recessive, and thus, options can be ranked.

## 3. Fuzzy ELECTRE Method

Suppose we have a MCDM problem where there are “*n*” options (*A*_1_ … *A*_*n*_) and “*m*” criteria (indices) *c*_1_ … *c*_*m*_ each option evaluated in proportion to *m* criteria. All determined values in proportion to criteria are indicated by a decision matrix called matrix S and weight vector *w* = (*w*_1_ … *w*_*n*_) where sum is ∑_*j*=1_^*m*^*w*_*j*_ = 1. The components are fuzzy numbers. Usually, in fuzzy MCDM problems, values of options in proportion to criteria and relative values are expressed as fuzzy numbers.

Step 1: fuzzy decision matrix
Suppose the fuzzy decision matrix and the fuzzy weight matrix are as follows:
  (30) $$\begin{array}{c} \begin{array}{c} \tilde{\;}\\ y=\left(\begin{array}{ccc} {\tilde{y}}_{11} & \cdots & {\tilde{y}}_{1m}\\ \vdots & \ddots & \vdots \\ {\tilde{y}}_{n1} & \cdots & {\tilde{y}}_{nm} \end{array}\right) \end{array}\text{,}\\ \tilde{w}=\left({\tilde{w}}_{1},\ldots ,{\tilde{w}}_{j},\ldots ,{\tilde{w}}_{m}\right)\text{.} \end{array}$$
Step 2: normalization
The matrix defined in the previous step is normalized as follows:
  (i) The criteria are positive profits:
    (31) $$\begin{array}{c} \left({\left(a_{ij}\right)}_{N},{\left(b_{ij}\right)}_{N},{\left(c_{ij}\right)}_{N}\right)=\left(\frac{a_{ij}-a_{j}^{\min}}{{∆}_{\min}^{\max}},\frac{b_{ij}-a_{j}^{\min}}{{∆}_{\min}^{\max}},\frac{c_{ij}-a_{j}^{\min}}{{∆}_{\min}^{\max}},\frac{d_{ij}-a_{j}^{\min}}{{∆}_{\min}^{\max}}\right){\left({\tilde{y}}_{ij}\right)}_{N}\text{.} \end{array}$$
  (ii) The criteria are expenditure:
    (32) $$\begin{array}{c} \left({\left(a_{ij}\right)}_{N},{\left(b_{ij}\right)}_{N},{\left(c_{ij}\right)}_{N}\right)=\left(\frac{a_{ij}-a_{j}^{\min}}{{∆}_{\min}^{\max}},\frac{b_{ij}-a_{j}^{\min}}{{∆}_{\min}^{\max}},\frac{c_{ij}-a_{j}^{\min}}{{∆}_{\min}^{\max}}\right),i=1,\ldots ,n\text{.} \end{array}$$
If it is a trapezoidal number, for normalizing, we should do as follows:
  (33) $$\begin{array}{c} C_{j}^{\max}=\max C_{ij},C_{j}^{\max}=\max C_{ij},wherei=1,\ldots ,n\text{,}\\ \Delta_{\max}^{\min}=a_{j}^{\min}-c_{j}^{\max}\text{,}\\ \Delta_{\min}^{\max}=c_{j}^{\max}-a_{j}^{\min}\text{.} \end{array}$$
If it is a trapezoidal number, for normalizing, we should do as follows:
  (34) $$\begin{array}{c} {\left({\tilde{y}}_{ij}\right)}_{N}=\left({\left(a_{ij}\right)}_{N},{\left(b_{ij}\right)}_{N},{\left(c_{ij}\right)}_{N},{\left(d_{ij}\right)}_{N}\right)=\left(\frac{a_{ij}-a_{j}^{\min}}{{∆}_{\min}^{\max}},\frac{b_{ij}-a_{j}^{\min}}{{∆}_{\min}^{\max}},\frac{c_{ij}-a_{j}^{\min}}{{∆}_{\min}^{\max}},\frac{d_{ij}-a_{j}^{\min}}{{∆}_{\min}^{\max}}\right)\text{.} \end{array}$$
For expenditure criteria,
  (35) $$\begin{array}{c} {\left({\tilde{y}}_{ij}\right)}_{N}=\left({\left(a_{ij}\right)}_{N},{\left(b_{ij}\right)}_{N},{\left(c_{ij}\right)}_{N},{\left(d_{ij}\right)}_{N}\right)=\left(\frac{d_{ij}-d_{j}^{\max}}{{∆}_{\max}^{\min}},\frac{b_{ij}-a_{j}^{\min}}{{∆}_{\max}^{\min}},\frac{c_{ij}-a_{j}^{\min}}{{∆}_{\max}^{\min}},\frac{d_{ij}-a_{j}^{\min}}{{∆}_{\max}^{\min}}\right)\text{,}\\ d_{j}^{\max}=\max d_{ij\;}\text{,}\\ a_{j}^{\min}=\min a_{ij},i=1,\ldots ,n\text{,}\\ \Delta_{\min}^{\max}=d_{j}^{\max}-a_{j}^{\min}\text{,}\\ \Delta_{\max}^{\min}=a_{j}^{\min}-d_{j}^{\max}\text{.} \end{array}$$
Step 3: left and right number of fuzzy numbers
Left and right number of fuzzy numbers is obtained by the following formula:
  (36) $$\begin{array}{c} {\left(l_{s}\right)}_{ij}=\frac{{\left(b_{ij}\right)}_{N}}{1+{\left(b_{ij}\right)}_{N}-{\left(a_{ij}\right)}_{N}}\text{,} \end{array}$$
  (37) $$\begin{array}{c} {\left(R_{s}\right)}_{ij}=\frac{{\left(c_{ij}\right)}_{N}}{1+{\left(c_{ij}\right)}_{N}-{\left(b_{ij}\right)}_{N}}\text{.} \end{array}$$
For trapezoidal number,
  (38) $$\begin{array}{c} {\left(l_{s}\right)}_{ij}=\frac{{\left(b_{ij}\right)}_{N}}{1+{\left(b_{ij}\right)}_{N}-{\left(a_{ij}\right)}_{N}}\text{,}\\ {\left(R_{s}\right)}_{ij}=\frac{{\left(d_{ij}\right)}_{N}}{1+{\left(d_{ij}\right)}_{N}-{\left(c_{ij}\right)}_{N}}\text{.} \end{array}$$
Step 4: interval matrix
A matrix which its components are intervals is formed that has a left and right number for each fuzzy number, so we have two matrices:
  (39) $$\begin{array}{c} \left[\left(L_{s},R_{s}\right)=\left[\begin{array}{ccc} {\left[\left(L_{s},R_{s}\right)\right]}_{11} & \cdots & {\left[\left(L_{s},R_{s}\right)\right]}_{1m}\\ \vdots & \ddots & \vdots \\ {\left[\left(L_{s},R_{s}\right)\right]}_{n1} & \cdots & {\left[\left(L_{s},R_{s}\right)\right]}_{nm} \end{array}\right]\right]\text{,} \end{array}$$
  (40) $$\begin{array}{c} {\left[\left(L_{s},R_{s}\right)\right]}_{{\left.\tilde{\left(w\right.}\right)}_{N}}=\left({\left[\left(L_{s},R_{s}\right)\right]}_{1}\ldots {\left[\left(L_{s},R_{s}\right)\right]}_{j}\ldots {\left[\left(L_{s},R_{s}\right)\right]}_{m}\right)\text{.} \end{array}$$
A matrix from *Y*'s, decision matrix and a matrix from *W*'s, weight matrix.
Step 5: multiplying the normalized matrixes
Multiplying the normalized matrix in the normalized weight and forming the weighted normal matrix.
Step 6: specifying concordant and discordant criteria
For each pair of options *k*, *e*(*k*, *e* = 1,2,…, *m*), criteria set *j* ∈ {1,…, *m*} are divided into concordance and discordance subsets. Concordance set is the criteria set where option *k* is superior in proportion to option *e* and its complement set is the discordance set. The set of concordant criteria for positive and negative criteria is defined as follows:
  (41) $$\begin{array}{c} S_{ke}=\left\{j|v_{kj}\geq v_{ej}\right\}\text{,} \end{array}$$
  (42) $$\begin{array}{c} S_{ke}=\left\{j|v_{kj}\geq v_{ej}\right\}. \end{array}$$
The set of discordant criteria for positive and negative criteria is defined as follows:
  (43) $$\begin{array}{c} I_{ke}=\left\{j|v_{kj}<v_{ej}\right\}\text{,} \end{array}$$
  (44) $$\begin{array}{c} I_{ke}=\left\{j|v_{kj}<v_{ej}\right\}\text{.} \end{array}$$
Step 7:
The concordance matrix is a square matrix which its dimension is the number of options. Each of the elements of this matrix is called the index of concordance between the two options. The value of this index is obtained from the sum of the weightings of the criteria that exist in the concordance set. In other words, for calculating the index of concordance, options *k*, *e* should be compared, and its value is obtained from the sum of criteria where option *k* has the advantage to option *e*. In mathematical terms, the index of concordance is obtained from the following equation:
  (45) $$\begin{array}{c} C_{ke}=\frac{\sum_{j\epsilon s_{ke}}w_{j\;}}{\sum_{j=1}w_{j}}\text{.} \end{array}$$
In the set of normalized weights, ∑_*j*=1_*w*_*j*_ is equal to one so
  (46) $$\begin{array}{c} C_{ke}=\underset{j\epsilon s_{ke}}{\sum }w_{j}\text{.} \end{array}$$
The concordant index indicates the degree of *s* superiority option *k* has over option *e*, and the value varies from zero to one. By calculating the concordant index for all the pairs of options, one can define the concordance matrix as follows, and in general, this matrix is not symmetrical.
  (47) $$\begin{array}{c} \left[\begin{array}{ccc} -C_{12} & \cdots \cdots & C_{1m}\\ C_{m1} & \cdots \cdots & C_{m\left(m-1\right)-} \end{array}\right]\text{.} \end{array}$$
Step 8: determining the discordance matrix
Discordance matrix is a square matrix in which its dimension is the number of options. Each of the elements of this matrix is called the index of discordance between the two options. The value of this index is obtained from the following equation [28]:
  (48) $$\begin{array}{c} d_{ke}=\frac{\max_{j\epsilon I_{ke}}\left|v_{kj}-v_{ej}\right|}{\max_{j\epsilon J}\left|v_{kj}-v_{ej}\right|}\text{.} \end{array}$$
The value of the discordance index varies from zero to one. By calculating the discordance index for all option pairs, the discordance matrix can be defined as follows. In general, this matrix is not symmetric.
  (49) $$\begin{array}{c} D=\left[\begin{array}{ccc} - & d_{12}\ldots \text{.} & d_{1m}\\ d_{21} & -\ldots \ldots & d_{2m}\\ d_{m1} & \ldots \ldots \ldots d_{m\left(m-1\right)} & - \end{array}\right]\text{.} \end{array}$$
The information in the concordance matrix has major differences from the information in the discordance matrix, and in fact, this information is complimentary. Differences between weights are obtained by the concordance matrix, whereas the difference between the specified values is obtained by the discordance matrix.
Step 9: creating concordance matrix
In step 9, the way to calculate concordance is explained. At this point, a certain value is specified by the concordant index, which is called the threshold of concordance and is denoted by d̅ threshold of concordance is obtained by averaging the indices of concordance (elements of concordance matrix). In mathematical terms, the value of the concordant threshold is calculated from the following equation:
  (50) $$\begin{array}{c} \bar{d}=\overset{m}{\underset{k=1}{\sum }}\overset{m}{\underset{e=1}{\sum }}\frac{d_{ke}}{m\left(m-1\right)}\text{.} \end{array}$$
Concordance dominance matrix (*f*) is formed by the value of the concordance threshold. If the obtained number is greater than $\bar{d\;}\text{.}$, the *k* option superiority over *e* is acceptable; otherwise, *k* has no advantage over the *e* option. Thus, elements of the concordance dominance matrix are obtained from the following equation:
  (51) $$\begin{array}{c} f_{ke}=\left\{\begin{array}{cc} 1\text{,} & d_{ke}\leq \bar{d,}\\ 0\text{,} & d_{ke}>\bar{d}\text{.} \end{array}\right. \end{array}$$
Step 10: creating discordance dominance matrix
Discordance dominance matrix (*G*) is formed as the concordance dominance matrix. For this purpose, the discordance threshold d^®^ is calculated from the averaging of the discordant indices (elements of the discordance matrix). In mathematical terms, the value of the discordance threshold is calculated by the (50) equation. As stated in step 7, the lower the value of the discordance index, the better it is. Because it shows the superiority of option *k* over *e*. The matrices of the discordance dominance matrix *G* are calculated as (51) equation. Each member of the *G* matrix also indicates the dominance relationship between the options.
Step 11: Creating final dominance matrix
The final dominance matrix *H* is obtained by multiplying each element of the dominance matrix of *F* by its corresponding element of the discordance dominance matrix *G*.
  (52) $$\begin{array}{c} h_{ke}=f_{ke}g_{ke}\text{.} \end{array}$$
Step 12: Choosing best option

The final dominance matrix *H* gives a detailed description of options. For example, if the value of ℎ is equal, it means that the superiority of the option *k* over *e* is acceptable in both concordant and discordant cases (i.e., the advantage is greater than the threshold of concordance, and the disagreement or weakness is lower than the threshold of discordance). However, the option *k* still has the chance to be dominated by other options. An option should be chosen that is more dominant than submissive, and thus, the options can be ranked.

## 4. Numerical Example

**Example 1 .**

Evaluation of catering services can be a new and growing industry in the new Turkey. Catering companies in Turkey must be very competitive. Their customers often change their catering contractor because it is easy to replace them when a complaint is made or a mismatch occurs, and there are many companies in the sector [29]. In this section, the method is applicable to a real industrial case, and the file is belonging to one of the textile companies operating in Denizli, Turkey. The problem of choosing food from this textile company has been solved through the fuzzy ELECTRE method. It has six criteria, health (C_1_), resources (C_2_), meat flavour and variety (C_3_), quality of service (C_4_), price (C_5_), and quality of structure (C_6_). There are 5 options to choose the best one. The table corresponding to this problem and their limits are given in Tables 1 and 2. By using the new method, we find out the best option.

Left and right number of fuzzy numbers is obtained by (36) (37) formula.

The data in Table 3 are obtained from formula (40). After that, the set of concordant criteria for positive and negative criteria is obtained from the (41), (42), (43), and (44) formulas. Its results are shown in Table 4.

In the continuation of the work, by considering Table 4, the values of the concordance matrix and discordance dominance matrix are obtained by using relations (45) and (48), and the results are shown in Tables 5 and 6.

The final dominance matrix is obtained by multiplying each element of the dominance matrix by its corresponding element of the incompatibility dominance matrix as shown in Table 7.

Finally, by comparing the two uptrends and downtrends, the final ranking of the options is as follows:

(53) $$\begin{array}{c} A_{1}>A_{2}>A_{4}=A_{5}>A_{3}\text{.} \end{array}$$

The final results obtained from the method presented are the same as the results of the research of Aytac et al. The technique used to find the desired results is acceptable.

**Example 2 .**

Look at the example given by Chen and Hwang [30], where a country wants to buy fighter jets, six criteria must be considered: maximum speed (C_1_), range of ships (C_2_), maximum loading (C_3_), price (C_4_), reliability (C_5_), and maneuverability (C_6_). Four types of fighter jets should be considered that match these criteria.  Table 8 shows the fuzzy correction matrix.  Table 9 shows the left and right scores of each alternative, according to each criterion and the left and right scores of each criterion.

Left and right number of fuzzy numbers is obtained by (36), (37) formula. The data in Table 10 are obtained from relationship (40). After that, the set of concordant criteria for positive and negative criteria is obtained from the (41), (42), (43), (44).

Then, the next steps are performed as in the previous example, and the final dominance matrix is obtained by multiplying each element of the dominance matrix by its corresponding element of the incompatibility dominance matrix. Its results are shown in Table 11.

Finally, by comparing the two uptrends and downtrends, the final ranking of the options is as follows:

(54) $$\begin{array}{c} A_{3}>A_{1}>A_{4}>A_{2}. \end{array}$$

This result is completely consistent with the result obtained by Hadi and Mokhtari [25] who solved it by the fuzzy TOPSIS method.

## 5. Conclusion

In this paper, the left and right intervals are used for the first time in the approximate dominance method. Due to the problems in the ELECTRE method, left and right intervals have been used for the first time in this article. In fuzzy multi-criteria decision-making problems, it is a difficult task to rank the options based on the criteria obtained with numbers between [0,1]..In such a situation, ranking the options according to the criteria (criteria weight) of interval-value fuzzy numbers is used. There are many solutions to solve these problems in solving fuzzy-interval MCDM problems. The value of the best option does not necessarily have the farthest distance to the worst option and the closest distance to the best option. On the other hand, the interval method has problems such as monotony and interdependence, so we try to improve and rank the ranking using the approximate dominance method. In the approximate dominance method, we compare the options with each other according to the criteria. The methods before this method were all one-dimensional, but the ELECTRE method is the first method in which we compare each option to each criterion. On the other hand, the interval method is a dependent method, so the approximate dominance method eliminates this dependence and makes the interval method more practical. The fuzzy method, based on left and right scores, introduces the concept of set maximization and set minimization to determine the sorting value of each fuzzy number and uses these values to determine the number of fuzzy numbers. The method of approximate dominance (elimination and selection method consistent with reality) is one of the most popular ranking methods in the world. In this method, the options are compared with each other in pairs, and the dominant and weak options (dominant and defeated) are identified, and then, the weak and defeated options are eliminated. In this research, we present a way to solve these interval-valued fuzzy MCDM problems to solve this problem as much as possible and use this method to rank the options. Here, we try to expand the ELECTRE method by using the terms compatibility and noncompliance and use a new idea to solve such problems. Therefore, we try to express the idea of correcting compatibility and incompatibility issues.

## Figures and Tables

**Table 1:** Fuzzy decision matrix.

	*c*_1_	*c*_2_	*c*_3_	*c*_4_	*c*_5_	*c*_6_
*W*	(0.533, 0.733, .0.933)	(0.4, 0.6, 0.8)	(0.533, 0.733, .0933)	(0.467, 0.667, 0.867)	(0.4, 0.6, 0.8)	(0.333, 0.533, 0.733)
*A *_1_	(0.538, 0.769, 1)	(0.538, 0.769, 1)	(0.571, 0.786, 1)	(0.5, 0.714, 0.929)	(0.154, 0.385, 0.615)	(0.417, 0.667, 0.917)
*A *_2_	(0.308, 0.538, 0.769)	(0.385, 0.615, 0.846)	0.571, 0.786, 1)	(0.571, 0.786, 1)	(0.231, 0.462, 0.692)	(0.333, 0.583, 0.833)
*A *_3_	(0.077, 0.308, 0.538)	(0.308, 0.538, 0.769)	(0.429, 0.643, 0.857)	(0.286, 0.5, 0.714)	(0.538, 0.769, 1)	(0.35, 0.5, 0.75)
*A *_4_	(0.308, 0.538, 0.769)	(0.385, 0.615, 0.846)	(0.143, 0.357, 0.571)	(0.5, 0.714, 0.929)	(0.231, 0.462, 0.692)	(0.333, 0.583, 0.833)
*A *_5_	(0.462, 0.692, 0.923)	(0.538, 0.769, 1)	(0.286, 0.5, 0.714)	(0.286, 0.5, 0.714)	(0.308, 0.538, 0.769)	(0.5, 0.75, 1)

**Table 2:** Left and right normalized scores.

	*c*_1_	*c*_2_	*c*_3_	*c*_4_	*c*_5_	*c*_6_
*W*	[0.6108, 0.7775]	[0.5000, 0.6667]	[0.6108, 0.7775]	[0.5558, 0.7775]	[0.5000, 0.6667]	[0.4442, 0.6108]
*A *_1_	[0.6247, 0.8123]	[0.6247, 0.8123]	[0.6469, 0.8237]	[0.5881, 0.7646]	[0.3127, 0.5000]	[0.5336, 0.7336]
*A *_2_	[0.4374, 0.6247]	[0.5000, 0.6872]	[0.4666, 0.8237]	[0.4669, 0.8237]	[0.3753, 0.5626]	[0.4664, 0.6664]
*A *_3_	[0.2502, 0.4374]	[0.4374, 0.6247]	[0.3103, 0.7059]	[0.4186, 0.5881]	[0.6247, 0.8123]	[0.6247, 0.6000]
*A *_4_	[0.4373, 0.6264]	[0.5000, 0.6917]	[0.2940, 0.4703]	[0.5881, 0.7646]	[0.3753, 0.5626]	[0.4664, 0.6664]
*A *_5_	[0.5626, 0.7497]	[0.6246, 0.8123]	[0.4111, 0.5881]	[0.4111, 0.5881]	[0.4374, 0.6247]	[0.6000, 0.8000]

**Table 3:** Left and normalized weighted right scores.

	*c*_1_	*c*_2_	*c*_3_	*c*_4_	*c*_5_	*c*_6_
*A*_1_	[0.3816, 0.6317]	[0.3123, 0.5415]	[0.3951, 0.6404]	[0.3269, 0.5524]	[0.1563, 0.3333]	[0.2370, 0.4480]
*A*_2_	[0.2187, 0.4857]	[0.2500, 0.4581]	[0.2851, 0.6404]	[0.2595, 0.5951]	[0.1877, 0.3750]	[0.2071, 0.4070]
*A*_3_	[0.1529, 0.3400]	[0.2187, 0.6164]	[0.1895, 0.4311]	[0.2325, 0.4250]	[0.3123, 0.5415]	[0.2774, 0.3664]
*A*_4_	[0.2671, 0.4870]	[0.2500, 0.4611]	[0.1795, 0.3657]	[0.3269, 0.5524]	[0.1877, 0.3750]	[0.2071, 0.4070]
*A*_5_	[0.3437, 0.5829]	[0.3123, 0.5415]	[0.2510, 0.4572]	[0.0.2284, 0.4032]	[0.2187, 0.4164]	[0.2665, 0.4886]

**Table 4:** Concordance matrix.

Compare options	Concordance criteria	Discordance criteria
*A*_2_ *toA*_1_	*C*_1_, *C*_2_, *C*_3_, *C*_5_, *C*_6_	*C*_4_
*A*_3_ *toA*_1_	*C*_1_, *C*_2_, *C*_3_, *C*_4_, *C*_5_, *C*_6_	—
*A*_4_ *toA*_1_	*C*_1_, *C*_2_, *C*_3_, *C*_4_, *C*_5_, *C*_6_	—
*A*_5_ *toA*_1_	*C*_1_, *C*_2_, *C*_3_, *C*_4_, *C*_5_	*C*_6_
*A*_1_ *toA*_2_	*C*_4_	*C*_1_, *C*_2_, *C*_3_, *C*_5_, *C*_6_
*A*_3_ *toA*_2_	*C*_1_, *C*_2_ , *C*_5_, *C*_6_	*C*_3_, *C*_4_
*A*_4_ *toA*_2_	*C*_3_, *C*_4_, *C*_5_, *C*_6_	*C*_1_, *C*_2_
*A*_5_ *toA*_2_	*C*_3_, *C*_4_, *C*_5_	*C*_1_, *C*_2_, *C*_6_
*A*_1_ *toA*_3_	—	*C*_1_, *C*_2_, *C*_3_, *C*_4_, *C*_5_, *C*_6_
*A*_2_ *toA*_3_	—	*C*_1_, *C*_2_, *C*_3_, *C*_4_, *C*_5_, *C*_6_
*A*_4_ *toA*_3_	*C*_3_	*C*_1_, *C*_2_, *C*_4_, *C*_5_, *C*_6_
*A*_5_ *toA*_3_	*C*_4_	*C*_1_, *C*_2_, *C*_3_, *C*_5_, *C*_6_
*A*_1_ *toA*_4_	*C*_4_, *C*_5_	*C*_1_, *C*_2_, *C*_3_, *C*_6_
*A*_2_ *toA*_4_	*C*_1_, *C*_2_ , *C*_5_, *C*_6_	*C*_3_, *C*_4_
*A*_3_ *toA*_4_	*C*_1_, *C*_2_ , *C*_4_, *C*_5_, *C*_6_	*C*_3_
*A*_5_ *toA*_4_	*C*_2_ , *C*_4_ , *C*_6_	*C*_1_, *C*_3_, *C*_6_
*A*_1_ *toA*_5_	*C*_2_ , *C*_6_	*C*_1_, *C*_3_, *C*_4_, *C*_5_
*A*_2_ *toA*_5_	*C*_1_, *C*_2_ , *C*_5_	*C*_3_, *C*_4_, *C*_6_
*A*_3_ *toA*_5_	*C*_1_, *C*_2_, *C*_3_, *C*_6_	*C*_4_, *C*_5_
*A*_4_ *toA*_5_	*C*_1_, *C*_2_, *C*_3_, *C*_6_	*C*_4_, *C*_5_

**Table 5:** Concordance matrix $F\;\left(\bar{C}=\left[34.0068/20,43.324/20\right]=\left[1.70034,2.166\right]\right)$.

	*A *_1_	*A *_2_	*A *_3_	*A *_4_	*A *_5_
*A *_1_	—	1	1	1	1
*A *_2_	0	—	1	1	1
*A *_3_	0	0	—	0	0
*A *_4_	0	0	1	—	0
*A *_5_	0	0	1	1	—

**Table 6:** Discordance dominance matrix $\left(\bar{d}=\left[13.7994/20\right]=\left[0.68997\right]\right)$.

	*A *_1_	*A *_2_	*A *_3_	*A *_4_	*A *_5_
*A *_1_	—	1	1	1	1
*A *_2_	1	—	0	1	1
*A *_3_	0	0	—	0	0
*A *_4_	0	0	1	—	1
*A *_5_	0	0	1	0	—

**Table 7:** Total matrix.

	The number of dominance	The number of subservience	Discord
*A *_1_	4	0	4
*A *_2_	2	1	1
*A *_3_	0	3	−3
*A *_4_	1	2	−1
*A *_5_	1	2	−1

**Table 8:** Fuzzy decision matrix.

	*W*	*A*_1_	*A*_2_	*A*_3_	*A*_4_
*C*_1_	(0.60, 0.68, 0.75)	2.00	2.5	1.8	2.20
*C*_2_	(0.40, 0.50, 0.60)	1500	2700	2000	1800
*C*_3_	(0.40, 0.50, 0.60)	20000	18000	21000	20000
*C*_4_	(0.40, 0.05, 0.60)	5.50	6.5	4.5	5.00
*C*_5_	(0.75, 0.83, 0.90)	(0.3, 0.5, 0.7)	(0.1, 0.2, 0.3)	(0.7, 0.8, 0.9)	(0.3, 0.5, 0.7)
*C*_6_	(0.90, 0.95, 1.00)	(0.9, 0.95, 1)	(0.3, 0.5, 0.7)	(0.7, 0.8, 0.9)	(0.3, 0.5, 0.7)

**Table 9:** Left and right normalized scores.

	*c*_1_	*c*_2_	*c*_3_	*c*_4_	*c*_5_	*c*_6_
*W*	[0.41, 0.52]	[0.14, 0.29]	[0.14, 0.29]	[0.14, 0.29]	[0.63, 0.74]	[0.85, 0.92]
*A *_1_	[0.29, 0.29]	[0.00, 0.00]	[0.67, 0.67]	[0.50, 0.50]	[0.40, 0.60]	[0.87, 0.93]
*A *_2_	[1.00, 1.00]	[1.00, 1.00]	[0.00, 0.00]	[0.00, 0.00]	[0.11, 0.22]	[0.22, 0.44]
*A *_3_	[0.00, 0.00]	[0.42, 0.42]	[1.00, 1.00]	[1.00, 1.00]	[0.78, 0.89]	[0.63, 0.75]
*A *_4_	[0.57, 0.57]	[0.25, 0.25]	[0.67, 0.67]	[0.75, 0.75]	[0.40, 0.60]	[0.22, 0.44]

**Table 10:** Left and normalized weighted right scores.

*c*_1_	*c*_2_	*c*_3_	*c*_4_	*c*_5_	*c*_6_
[0.119, 0.151]	[0.000, 0.000]	[0.094, 0.194]	[0.070, 0.145]	[0.252, 0.444]	[0.730, 0.850]
[0.410, 0.520]	[0.140, 0.290]	[0.000, 0.000]	[0.000, 0.000]	[0.069, 0.163]	[0.187, 0.405]
[0.000, 0.000]	[0.059, 0.122]	[0.140, 0.290]	[0.140, 0.290]	[0.491, 0.659]	[0.536, 0.690]
[0.234, 0.296]	[0.035, 0.0725]	[0.094, 0.1943]	[0.105, 0.217]	[0.252, 0.444]	[0.187, 0.405]

**Table 11:** Total matrix.

	The number of dominance	The number of subservience	Discord
*A *_1_	2	0	2
*A *_2_	1	1	0
*A *_3_	3	0	3
*A *_4_	2	1	1

## Data Availability

The data used to support the findings of this study are available from the corresponding author upon request.
